# The Molecular Blueprint for Chronic Obstructive Pulmonary Disease (COPD): A New Paradigm for Diagnosis and Therapeutics

**DOI:** 10.1155/2023/2297559

**Published:** 2023-12-21

**Authors:** Ilma Shakeel, Anam Ashraf, Mohammad Afzal, Sukhwinder Singh Sohal, Asimul Islam, Syed Naqui Kazim, Md. Imtaiyaz Hassan

**Affiliations:** ^1^Department of Zoology, Aligarh Muslim University, Aligarh, Uttar Pradesh 202002, India; ^2^Centre for Interdisciplinary Research in Basic Sciences, Jamia Millia Islamia, Jamia Nagar, New Delhi 110025, India; ^3^Respiratory Translational Research Group, Department of Laboratory Medicine, School of Health Sciences, College of Health and Medicine, University of Tasmania, Launceston, Tasmania 7248, Australia

## Abstract

The global prevalence of chronic obstructive pulmonary disease (COPD) has increased over the last decade and has emerged as the third leading cause of death worldwide. It is characterized by emphysema with prolonged airflow limitation. COPD patients are more susceptible to COVID-19 and increase the disease severity about four times. The most used drugs to treat it show numerous side effects, including immune suppression and infection. This review discusses a narrative opinion and critical review of COPD. We present different aspects of the disease, from cellular and inflammatory responses to cigarette smoking in COPD and signaling pathways. In addition, we highlighted various risk factors for developing COPD apart from smoking, like occupational exposure, pollutants, genetic factors, gender, etc. After the recent elucidation of the underlying inflammatory signaling pathways in COPD, new molecular targeted drug candidates for COPD are signal-transmitting substances. We further summarize recent developments in biomarker discovery for COPD and its implications for disease diagnosis. In addition, we discuss novel drug targets for COPD that could be explored for drug development and subsequent clinical management of cardiovascular disease and COVID-19, commonly associated with COPD. Our extensive analysis of COPD cause, etiology, diagnosis, and therapeutic will provide a better understanding of the disease and the development of effective therapeutic options. In-depth knowledge of the underlying mechanism will offer deeper insights into identifying novel molecular targets for developing potent therapeutics and biomarkers of disease diagnosis.

## 1. Introduction

Chronic obstructive pulmonary disease (COPD) is a common breathing difficulty caused by the blockage of airflow and other associated breathing problems. It includes chronic bronchitis and emphysema. Airflow limitations are primarily due to remodeling and inflammation of the airways, which is often associated with the destruction of the parenchyma and the development of emphysema. The statistics in 2020 reported COPD as the third leading cause of death worldwide [1].

The interaction between different factors, including environmental and genetic factors, contributes to COPD risk. The most important and most common risk factor for COPD is cigarette smoking. In contrast, other risk factors include occupational/workplace exposure, air pollution, coal dust, asthma, airway hyper-responsiveness, and genetic predispositions [2–4]. Various pulmonary symptoms contribute to a progressive limitation in the airflow of COPD patients, including emphysema and small airway disease (SAD). SAD, called obstructive bronchitis, involves airway inflammation with increased mucus production, peribronchial fibrosis, and remodeling of airway walls [5]. Spirometry is used for the assessment of the degree of airflow limitation. According to global initiative for chronic obstructive lung disease (GOLD) criteria, the severity of COPD is classified spirometrically using the FEV1/FVC ratio [6, 7]. Other grading systems include BODE, where B is the body mass index, O is the airflow obstruction, D is the dyspnoea, and E is the exercise tolerance [8].

Many diseases co-occur with COPD and increase the severity and mortality of the patients, including cardiovascular diseases, malnutrition, osteoporosis, skeletal muscle dysfunction, anaemia, anxiety, depression, and increased gastroesophageal refluxes. The limitation of airflow in patients with COPD increases the likelihood of the patients developing pulmonary cancer over some time. Additionally, patients with COPD belong to the old age group, and the high prevalence of comorbidities requires more extensive medical care. Moreover, the risk of hospitalization and death increases, mainly due to severe airway obstruction [9]. Systemic inflammation in patients with COPD, together with activated inflammatory cells, raises the cytokine levels in the systemic circulation and increases oxidative stress. So, in the light of these researches, it was proposed recently to include the term “chronic systemic inflammatory syndrome” for diagnosing COPD [10].

Biomarkers are characteristics measured as indicators of normal biological processes, pathogenic processes, or responses to an exposure or intervention [11]. Biomarkers can be further categorized into various subtypes based on their relative utilization. It helps define the progression of the disease during pathogenesis. Biomarkers, combined with clinical symptoms, play an essential role in identifying the etiological origin and severity of the disease. Levels of biomarkers can be correlated toward response to therapy intervention, helping us assess the clinical evolution of the disease, and giving us insights into the potential complications that may arise. COPD pathogenesis majorly consists of overexpression of systemic inflammation markers and signaling pathways. Thus, determining these markers is one of the imperative and crucial directions in improving the diagnosis and management of COPD [12].

A multidisciplinary approach is required to optimize the therapeutic management of patients suffering from COPD [13]. Cessation of smoking, oxygen therapy, pharmacological therapy with glucocorticoids and bronchodilators, surgery, and pulmonary rehabilitation are the cornerstone of COPD management, making COPD a treatable and preventable disease [14]. Two types of therapies are used, including the therapy primarily centered in the lung, whereas the latter center shifts to a systemic inflammatory state.

In this review, we discussed the mediators of cellular signaling mechanisms in COPD, the risk factors involved in the progression of the disease, and different types of diagnostic biomarkers used to detect and confirm COPD. Here, we summarized the comorbid diseases with COPD and elaborated on the therapeutic perspectives of approved drugs and ongoing clinical trials. This study provides an extensive literature review followed by an in-depth and critical analysis of the state of the art and identifies challenges for future research.

## 2. Mediators of Cellular Signaling in COPD

COPD is a group of diseases that causes breathing-related issues and causes blockage of airflow. There are various cellular and inflammatory interactions caused by smoking cigarettes in COPD. Activation of various immunological cells, such as B-cells, T-cells, dendritic cells, macrophages, and neutrophils, and activation of epithelial cells, airway smooth muscle cells, and fibroblast cells results in the release of proteases, chemokines, and cytokines and hence causing COPD [15].

### 2.1. Role of NF-*κ*B Pathway in COPD

Various canonical and noncanonical pathways play an essential role in the development and pathogenesis of COPD by overexpressing pro-inflammatory factors, causing chronic inflammation in the lungs. Furthermore, NF-*κ*B-regulated genes such as adhesion molecules, cytokines, matrix metalloproteinases (MMPs), antiapoptotic factors, and angiogenic factors are associated with the progression of the disease. Thus, the first line of therapy in lung cancer and COPD is the downregulation of NF-*κ*B activation [16].

### 2.2. Role of Adaptive Immune Response and Immune Sculpting

The main features of chronic inflammation in COPD patients are the accumulation of CD4+-T, CD8+-T cells, B-cells, dendritic cells, macrophages, neutrophils, and eosinophils in the small airways [5]. Infiltration of these inflammatory immune cells is associated with the severity of COPD disease. The central role of these inflammatory immune cells in COPD patients is the release of granzymes, proteinases, perforins, and oxidants, which destroy the walls and cause the hypersecretion of mucus [17].

### 2.3. Role of Adhesion Molecules

Integrins (heterodimeric transmembrane receptors) are involved in various cellular functions and lung inflammation. The expression of integrin avb6 (localized in epithelial cells) increases during injury and inflammation of the lungs [16]. Moreover, in COPD patients, there is an upregulation of TGF-*β*1 protein and mRNA in both the airways and alveolar epithelium cells. TGF-*β*1 mRNA levels correlate positively with the history of smoking and the degree of obstruction in the small airways, suggesting the proremodeling, profibrogenic, and cell-specific roles of TGF-*β* in the patients of COPD [16].

### 2.4. Role of Hypoxia or Angiogenesis

Hypoxia induces lung inflammation either by influencing the expression of pro-inflammatory genes or by activating transcription factors. In patients with COPD, damaged alveolar capillaries and progressive airflow limitations lead to reduced oxygen transport and cause alveolar hypoxia. Furthermore, hypoxia-inducible factor activation induces vascular endothelial growth factor (VEGF) transcription and increases angiogenesis. Thus, clinically, oxygen therapy can be significant in providing temporary relief in hypoxemic COPD patients. Interestingly, chronic oxygen therapy may result in oxidative cellular injury, resulting in aggravation of pulmonary inflammation and cell mortality. VEGF expression is also increased in chronic bronchitis patients [18], suggesting that VEGF has a paradoxical role in the airspaces and bronchi of COPD patients.

### 2.5. Role of Matrix Metalloproteinases (MMPs)

Emphysema is caused by the shift between the balance of proteinases and antiproteinases (shifts toward proteinases), including MMPs and elastase in the lungs' activated epithelial cells and inflammatory cells. Due to the defective tissue repair and degradation of ER membrane protein complex (EMC) by MMPs, the lungs' structural cells undergo apoptosis and lose their attachment. Additionally, the chemotactic activity of EMC fragments attracts inflammatory cells into the lungs, which results in further progression of emphysema in the mice model [19].

## 3. Risk Factors of COPD

The interaction between different factors, including environmental and genetic factors, contributes to COPD risk. Comorbid diseases can also affect the interaction between different factors. Risk factors for COPD are summarized in Figure 1.

### 3.1. Smoking Tobacco

Smoking tobacco is the leading causative factor of COPD worldwide. According to the estimate of WHO, 73% of COPD mortalities are present in high-income countries, whereas only 40% of COPD mortalities are present in low or middle-income nations [20]. Genes or genetics have a significant role in this relationship, as all smokers do not develop COPD. However, ∼50% of smokers develop COPD in their later life [21]. Smoking during the gestational period can negatively affect fetal lung growth and, therefore, results in the development of various lung diseases [22].

Cessation of tobacco smoking is the most effective intervention in preventing COPD progression, thus reducing morbidity and increasing the survivability of the patients [23]. Apart from tobacco, marijuana smoking has also been linked to various respiratory symptoms, but its direct relation to COPD development is unknown [24].

### 3.2. Occupational Exposure

Factory workers are exposed to various workplace factors, including dust, mist, fumes, vapors, and various chemicals, which is also a factor in causing COPD in factory workers or associated people [25]. In an estimate, it was shown that in the USA, 19.2% of COPD cases were attributed to exposure to workplace factors, out of which 31.1% cases were the proportion of being never smokers in their life and still develop COPD [26]. Another report showed that people diagnosed with chronic bronchitis or COPD were twice as likely to have previous workplace exposure to fumes, gases, vapors, and dust [27].

Due to less stringent laws in low and middle-income countries, work exposure to fumes and dust is remarkably greater than in high-income countries, where laws are comparatively more stringent. Hence, workplace exposure is assumed to be an important risk factor for COPD.

### 3.3. Air Pollution

In poorly ventilated homes, cooking or heating exposes biomass fuels such as wood, animal dung, coal, straw, and crop residues. These are considered essential risk factors in COPD development, primarily in rural households. One of the reports from China suggests that the prevalence of COPD is twice or thrice times higher in never-smoker women in rural areas, where women have greater exposure to biomass smoke than urban women without such exposures [28]. According to the estimate of WHO, in low and middle-income countries, 35% of people develop COPD after exposure to biomass fuels and indoor smoke [20]. Furthermore, WHO also suggested that 36% of mortality from lower respiratory diseases is directly related to exposure to indoor smoke [20].

Apart from direct smoke exposure, second-hand smoke inhalation is another form of biomass smoke linked to various respiratory diseases. However, its direct relation to COPD is not known [29].

The risk attributes for COPD development from outdoor air pollutants are remarkably lesser than indoor air pollutants. According to an estimate by WHO, in higher income countries, only 1% of COPD cases are developed by urban air pollution, and only 2% in low and middle-income countries [20]. Outdoor air pollution, or simple air pollution, is linked to acute cardiopulmonary events and various respiratory infections essential in developing and progressing COPD.

### 3.4. Genetic Factors

The functioning of the lungs in offspring is complexly related to the parental lung functions [30]. Out of all offspring whose both parents lie in the lowest quintile group of lung functioning, 37% of the offspring lie in the lowest quintile group of lung function compared to their peers [30]. On the other hand, out of all offspring whose parents lie in the highest quintile group of lung functioning, 41% of the offspring lie in the highest quintile group of lung functioning compared to their peers [30].

Serine protease *α*1-antitrypsin deficiency is one of the best-known genetic factors linked to COPD. Serine protease *α*1-antitrypsin deficiency arises in 1%–3% of patients with COPD [31]. A low concentration of *α*1-antitrypsin, particularly in amalgam with tobacco smoking and other exposures, increases the probability of pan lobular emphysema [31].

Various studies show that several genes are involved in COPD, such as microsomal epoxide hydrolase 1 [32], tumor necrosis factor (TNF)*-α* [33], and transforming growth factor*-β*1 [34]. However, research is still under trial to examine the specific polymorphisms in the abovementioned genes for COPD development. A study by Zhou et al. [35] on the Chinese population shows that the genetic polymorphism in MIR5708 and MIR1208 is related to the susceptibility to COPD.

### 3.5. Infection

According to a review of *The Lancet*, most of the exacerbations of COPD are either due to viral infections or bacterial infections [36]. Various infections play an essential role in the development and progression of the disease. Early-life exposure to infections could make the individual susceptible to bronchiectasis and change the airways' responsiveness.

### 3.6. Aging

The age-related decline in pulmonary function is considered normal. With the increase in age, the prevalence, mortality, and morbidity of COPD also increase. The peak level of pulmonary function reaches young adulthood, which declines in the third or fourth decades of life [36]. However, some researchers have reported that in old age, people with a high level of pulmonary function live comparatively longer than those with lower pulmonary functions [37].

Aging is a natural process, where, at the cellular level, it includes various molecular and systemic mechanisms. In several studies, the role of specific senescence pathways, such as sirtuin family proteins and p-16, has become evident and is implicated in COPD and aging [38]. Various common DNA-level abnormalities, leucocyte response abnormalities, and inflammatory markers were increased both in COPD and aging [38].

In recent years, the prevalence of COPD has increased due to the demographic changes in the world's population, which are attributed to a good nutritional life, and, hence, the reduction and elimination of various infectious diseases in childhood. Therefore, falling in mortality rates are falling due to diseases that kill or eliminate younger people earlier, such as acute infections and cardiac diseases. This leads to a longer life expectancy in most of the world's population and increases the risk for several chronic medical conditions, including COPD [39].

### 3.7. Socioeconomic Status

Populations with lower socioeconomic status or the population who live in poverty have a higher risk of developing COPD and its related complications compared to their wealthier counterparts [40]. Poverty is considered a surrogate for poor access to health care, poor nutritional status, overcrowding (large family size), more exposure to occupational pollutants (such as, fumes, dust, mists, and chemicals), high rates of tobacco smoking (in low and middle-income countries), and early respiratory infections, and hence, increases the risk of COPD subsequently [40].

In the study by Eisner et al. [41], a consistent and significant inverse relation was observed between the outcomes of socioeconomic status and COPD, which may be used to validate the time and costs needed for the development, research, and implementation of the strategies to improve the health of COPD patients.

### 3.8. Gender

The role of gender in both the progression and development of COPD is highly controversial and is a topic of a great deal in the scientific community [42]. Earlier in men (due to occupational exposure and related patterns of tobacco smoking), COPD is considered far more frequent than in women of the same age [43]. However, lately, the prevalence of COPD has become equally likely in men and women of higher income countries where the habit of smoking tobacco is similar between the two sexes. Some studies showed that women are more likely to develop COPD than men. By giving equal exposure to smoking and the same environmental factors, researchers support the hypothesis that women are more susceptible to developing COPD than men [44].

## 4. Diagnostic Biomarkers for COPD

COPD is a diverse disease affecting multiple organs, establishing a systemic infection. Recently, studies have shifted their focus to biomarkers to illustrate the pathogenesis and progression of the disease. A detailed and systematic study on biomarkers can pave a new road to designing novel therapeutic targets for COPD [45]. Biomarkers can be defined fundamentally and straightforwardly as “A defining characteristic that is measured as an indicator of normal biological processes, pathogenic processes, or responses to an exposure or intervention” [11].

Biomarkers can be further categorized into various subtypes based on their relative utilization. Biomarkers help define the progression of the disease during pathogenesis. Biomarkers, combined with clinical symptoms, play a role in identifying the etiological origin and severity of the disease. Levels of biomarkers can be correlated toward response to therapy intervention, helping us assess the clinical evolution of the disease and giving us insights into the potential complications that may arise. Thus, studying these biomarkers will enable us to manage the disease better with better risk stratification. They may also guide us in assessing the effectiveness of clinical trials.

This review will discuss the different types of diagnostic biomarkers used to detect and confirm COPD. These biomarkers help identify the diseased population and aid us in redefining the disease classification. COPD pathogenesis majorly consists of overexpression of systemic inflammation markers and signaling pathways. Thus, determining these markers is one of the imperative and crucial directions in improving the diagnosis and management of COPD [12]. The following are the significant diagnostic biomarkers for the detection and management of COPD (Figure 2).

### 4.1. C-Reactive Protein

The overexpression of C-reactive protein (CRP) is known at the site of inflammation and infection, as it is an acute inflammatory protein. CRP is the predominant mediator of the acute phase response in an inflammatory event, primarily synthesized by IL-6-dependent hepatic biosynthesis [46]. The serum CRP levels in COPD patients were significantly higher than those of healthy subjects [47]. In COPD patients, the levels of CRP were directly associated with age and inversely related to hemoglobin levels. Studies have found that lung function indices such as dyspnea score, oxygen saturation, and 6-min walking distance (6MWD), potential COPD severity predictors, substantially correlate with CRP levels. Factors such as duration of the disease and BMI in COPD patients show no correlation with CRP levels [48].

Increased serum CRP baseline is more pronounced in COPD mortality than COPD hospitalization cases, consistently marking functional and metabolic damage in advanced COPD [49]. Thus, in the case of COPD exacerbation, CRP is used as a diagnostic biomarker, and for early mortality cases of COPD, it is used as a prognostic biomarker [50, 51]. CRP levels can also be used as an informative biomarker as they can demonstrate low-grade systemic inflammation [52]. Lately, studies have shown the association of serum CRP levels with several different outcomes, including COPD exacerbation [53].

### 4.2. Interleukin-6

Interleukin-6 (IL-6) plays a vital role in systemic inflammation of COPD patients, as it is a crucial pro-inflammatory cytokine [54]. In the stable and exacerbation phases of COPD patients, the circulatory level of IL-6 was higher than healthy controls [55]. Among the severity of COPD, the circulatory levels of IL-6 were found to be of significant difference, further defining that the level of IL-6 was higher in mild, moderate, severe, and very severe COPD patients [56].

The pro-inflammatory cytokine IL-6 can induce acute-phase proteins like CRP. Thus, the levels of CRP and IL-6 were correlated in COPD patients [57]. COPD exacerbations lead to overexpression of IL-6 in serum, which leads to a surge of plasma fibrinogen. Thus, acute COPD response can prime for stroke or coronary heart disease as comorbidity [58]. A recent finding has established a relation between the plasma level of IL-6 in malnutrition pathophysiology and low-weight COPD patients. The study has also elucidated the sensitivity of the serum level of IL-6 compared to other inflammatory factors in predicting COPD disease development in smokers [59].

IL-6 is the primary regulator in many inflammatory pathways contributing to disease progression. Thus, IL-6 can independently be a predictive power in determining mortality in a basic clinical model [60]. IL-6 serum levels have also been associated with poor physical function in COPD patients irrespective of age, gender, race, and body composition [61]. IL-6-driven inflammation may complicate COPD by contributing extensively to pulmonary hypertension, leading to increased morbidity of the disease [62]. We can summarize the systemic inflammatory process led by IL-6 in COPD patients coerced toward a progressive and persistent disease model with associated mortality and inconsistent physical performance [63].

### 4.3. Serum Amyloid A

Serum amyloid A (SAA) is a protein of the acute phase having numerous immunological functions. It involves various processes such as inflammatory reactions, lipid metabolism, and granuloma formation. It has an established role in autoimmune lung disease pathogenesis. SAA is used as a biomarker in various lung diseases such as COPD, obstructive sleep apnea (OSA) syndrome, asthma, lung cancer, and cystic fibrosis [64]. SAA has been identified as a novel blood biomarker for acute exacerbation of chronic obstructive pulmonary disease (AECOPD). Changes in SAA levels have shown higher sensitivity and specificity in defining AECOPD severity than other biomarkers like CRP. A significant increase in SAA levels above baseline predicts severe AECOPD [65]. For early detection and management of AECOPD, SAA-level determination is advantageous. It can help categorize the patients with the highest risk of respiratory failure. Biomarkers like IL-6 remain uninformative in severe cases of AECOPD [65].

Patients with AECOPD and COPD have inflammatory reactions and have high blood viscosity, thus showing significantly higher levels of SAA compared to the healthy control group. For the clinical diagnosis and treatment of AECOPD, SAA can be used as an effective index [66]. In the resolution phase of infection, the secretion of SAA becomes self-limiting and protective with a sharp fall. In the AECOPD, there is a steady rise in SAA levels elicited by coinfections [67]. Exhilarated levels of SAA are also associated with cardiovascular diseases, where COPD is a comorbidity. Exacerbation episodes lead to a dramatic increase in mortality related to cardiovascular events in COPD. SAA levels can very well anticipate future cardiovascular events; thus, SAA can be scrutinized as a predictor for frequent exacerbation phenotypes and a marker for comorbid cardiovascular disease [68].

### 4.4. Tumor Necrosis Factor

TNF is a potent cytokine that mediates inflammation and immune response. It recruits acute phase proteins, transcription factors, cell surface receptors, and cytokines [69]. TNF starts the production of interleukin cascade components when secreted excessively. It can also instigate the secretion of matrix metalloprotease 9, which contributes to lung emphysema, one of COPD's major symptoms [70]. Recently, a meta-analysis study has shown compelling results for a direct relationship between COPD and elevated TNF-*α* levels. Higher TNF-*α* level was found in COPD patients in comparison to healthy controls. It may also play a role in the progression and diagnosis of COPD, but its mechanism is still unknown and needs to be further explored [71].

In the pathophysiology of COPD, TNF-*α* tends to play a central role. Different cells, like alveolar macrophages and T-cells, produce TNF-*α* in response to various pollutants, including cigarette smoke [72]. Studies with animal models have shown the induction of pathological features of COPD, like emphysema and lung fibrosis, following elevated TNF-*α* levels [73]. The role of TNF-*α* during COPD is limited to enhancing inflammatory events and developing systemic inflammation within the respiratory tract, which manifests in cachexia in severe COPD patients. Thus, TNF-*α* is directly associated with the severity of the disease and its progression [74].

### 4.5. Fibrinogen

Fibrinogen is a soluble plasma glycoprotein majorly involved in blood coagulation reactions by converting thrombin into fibrin. It can increase significantly during acute phase stimulation in response to increased IL-6 production [75]. A deterioration in lung function can be associated with elevated plasma fibrinogen concentration, which increases the risk of developing COPD [76]. For exacerbation of COPD, elevated fibrinogen can act as an independent risk factor [77].

Fibrinogen is a glycoprotein with biological roles closely associated with cell adhesion, blood coagulation, phagocytosis, extension, proliferation, etc. [78]. The molecular weight of fibrinogen is the largest in available coagulogens, having structure chain-like asymmetric, and can increase the thickening of plasma, contributing to the formation of small pulmonary arterial thrombi and aggravating lung injury [79].

Food and Drug Administration (FDA), USA, and European Medicines Agency (EMA) have qualified plasma fibrinogen as a severity assessment COPD biomarker and qualified it as a drug development tool [80]. As issued by the FDA and EMA, circulating fibrinogen can be suggested as a biomarker for early warning. It can be a potent predictor of future susceptibility to develop COPD and its severity [81].

## 5. Comorbidities in COPD

Many diseases co-occur with COPD and hence increase the severity and mortality of the patients. The comorbid diseases could also affect the interaction between different environmental factors and their impact on the severity of the disease. Comorbid diseases of COPD are summarized in Figure 3.

### 5.1. COVID-19

Patients with preexisting COPD are susceptible to worsening the prognosis and progression of COVID-19 [82]. Meta-analysis studies on COVID-19 from December 2019 to March 2020 demonstrate that the severity of COVID-19 increases fourfold in patients with preexisting COPD [83, 84]. The analysis in China for comorbidities in 1,590 COVID-19-positive patients found that the odds ratio of COPD is about 2.681 (95% CI 1.424–5.048; *p*=0.002) for ICU patients, ventilators, or death, even after adjusting the smoking and age [84–87]. Furthermore, out of all severe cases, 62.5% of cases had a history of COPD, whereas, in comparison, only 15.3% of cases had a history of COPD in nonsevere cases. Additionally, out of the total fatalities, 25% of cases are COPD patients, whereas, in comparison, only 2.8% of COPD patients have survived.

Cellular serine protease (TMPRSS2) primes the envelope spike protein of SARS-CoV-2 and hence helps to facilitate the fusion of the SARS-CoV-2 virus with angiotensin-converting enzyme 2 receptor (ACE-2 receptor) in the cells and subsequently facilitates the cell entry [88, 89]. In COPD patients, the expression of ACE-2 was significantly elevated in bronchial epithelial cells compared to the control subjects [90]. However, it is interesting to note that the expression of ACE-2 alone has neither shown an increase in the severity of the disease nor an increase in its susceptibility. Moreover, in patients with predominantly small airway pathologies, ACE-2 expression is relatively low in the bronchial epithelium compared to the nasal epithelium. It has unexplained implications for the susceptibility of the disease [91].

### 5.2. Lung Cancer

COPD patients are three to four times more susceptible to developing pulmonary cancer than tobacco smokers with normal pulmonary functions [92]. Lung cancer is one of the significant causes of fatality in COPD patients, especially in patients with more severe diseases [93]. An increase in the prevalence of pulmonary cancer in patients with COPD is more likely associated with an increase in oxidative stress and inflammation in COPD patients [94]. NF-*κ*B activation might provide a link between lung cancer and inflammation [95]. By regulating the expression of various detoxifying enzymes, nuclear factor erythroid 2-related factor 2 (Nrf2) plays a vital role in defending against several carcinogens of tobacco inhalation. As COPD patients lack Nrf2, it might contribute to increasing the susceptibility of COPD patients to pulmonary cancers [96].

It is interesting to note that lung cancer is more common among patients with COPD who are never smokers and have never been exposed to tobacco inhalation in their entire life [97]. In females, the risk of getting lung cancer and COPD is greater, probably due to the hormone-stimulated metabolism of carcinogens in smoking tobacco [98].

### 5.3. Muscle Dysfunction and Malnutrition in COPD

Weakness in the skeletal muscles is one of the important systemic effects of COPD, often accompanied by the loss of fat-free mass (FFM) [99]. In normal males, 40%–50% of total body mass accounts for skeletal muscle. The turnover of proteins in skeletal muscle is a dynamic process involving balancing protein breakdown and protein synthesis. Moreover, in acute illnesses like sepsis and trauma, the loss of muscle mass due to the breakdown of muscle proteins is comparatively more significant. It occurs rapidly, whereas in chronic illnesses like COPD, the loss of muscle mass due to muscle protein breakdown is comparatively slower. Several studies demonstrate that in patients with COPD, the structure and function of skeletal muscles are altered. Several studies on humans indicate that the breakdown of skeletal muscle is evident in patients with COPD and is specific for muscle fiber type IIA/IIx [100].

Muscle wasting has a magical effect on morbidity in severe cases of COPD. Hence, it increases the risk of readmission to the hospital after an exacerbation and increases the need for mechanical ventilation support. Additionally, muscle wasting is considered a significant determinant of mortality in patients with COPD independently of smoking, BMI, and lung functions [101].

### 5.4. Diabetes

Several population studies indicated an increase in the prevalence of diabetes among patients with COPD, with a relative risk of 1.5–1.8 [9]. Even in patients with mild symptoms of COPD, the prevalence of diabetes is observed [9]. The mechanism behind this association is not precise. Furthermore, the relation between high doses of inhaled corticosteroids and the increased risk of diabetes is also doubtful. Patients with mild disease also have a high risk of diabetes. It is interesting to note here that asthma patients do not have the prevalence of diabetes. However, COPD does have it, suggesting an altogether different mechanism of inflammation in COPD compared to asthma.

Pro-inflammatory cytokines like IL-6 and TNF-*α*, induce insulin resistance by inhibiting the signals of insulin receptors, thereby increasing the risk of type-2 diabetes [102]. An increase in the concentration of plasma CRP, IL-6, and TNF-*α* are reported in metabolic syndromes, including cardiovascular diseases and insulin resistance [103]. These metabolic syndromes are also prevalent among patients with COPD, thus leading to the co-occurrence of cardiovascular diseases and diabetes with airway obstruction [103].

### 5.5. Osteoporosis

Multiple studies have shown that in patients with COPD, there is a very high prevalence of low bone mineral density (BMD) and osteoporosis, even in the milder stages of COPD disease [104]. In a study, 6,000 COPD patients were recruited for the large TORCH trial (toward a Revolution in COPD Health); among these, over half of the COPD patients have osteopenia or osteoporosis, which is determined by Dexa (dual-energy radiograph absorptiometry) [105]. In another study, there is a 75% prevalence of osteoporosis in patients with GOLD stage IV disease, and it has a strong correlation with the decrease in the level of FFM [106, 107].

It is interesting to note that the prevalence of osteoporosis is high in males and even higher in the case of females. At the same time, the incidences of nontraumatic and traumatic fractures are approximately similar in both sexes. Fractures due to vertebral compression are relatively widespread among patients with COPD, and this increase in kyphosis further reduces the functions of the lung [108].

### 5.6. Normocytic Anemia

Several studies have shown that the prevalence of anemia is very high among patients of COPD, ranging between 15% and 30% of total COPD patients, especially in patients with more severe disease conditions. In contrast, erythrocytosis (polycythemia) is comparatively rare, ranging about 6% [109, 110]. Hemoglobin level is independently and strongly associated with the increase in functional dyspnea, and decrease in exercise capacity, and hence, is an essential contributor to functional capacity and poor quality of life [111]. For chronic inflammation diseases, the anemia is usually of characteristic normochromic normocytic type, which appears to be due to resistance to the erythropoietin, whose concentration is elevated in these patients [112].

In a study, it was shown that the transfusion of blood improves exercise performance in anaemic COPD patients [113]. However, iron supplements show detrimental effects as iron cannot be utilized correctly and may increase systemic oxidative stress.

### 5.7. Obstructive Sleep Apnea

The condition during sleep where the upper airways collapse repetitively is known as obstructive sleep apnea (OSA). According to an estimate, 20% of OSA patients also have underlined COPD conditions. Of their counterparts, 10% of COPD patients have the severity of the disease independent of OSA [114]. OSA and COPD patients share many common comorbidities, including cardiac failure, endothelial dysfunction, metabolic syndrome, and diabetes [115]. According to some recent research, it is evident that patients with OSA have systemic inflammation, upper airway inflammation, and oxidative stress [116].

### 5.8. Depression

Due to the physical limitations of COPD patients, they are more often isolated and unable to engage themselves in various social activities. So, it is not surprising to see an increase in the prevalence of depression and anxiety in patients with COPD, and depression and anxiety appear to be more prevalent in COPD than in any other chronic disorder. The symptoms of depression and anxiety are often confused with the symptoms of COPD; hence, they remain undiagnosed and untreated in various clinical practices. Clinically relevant symptoms of depression are estimated to occur in about 10%–18% of all patients. However, among the clinically stable outpatients with COPD, about 19%–42% prevalence is seen for major depression, which requires therapeutical interventions [117, 118]. Depression cannot be diagnosed with any standardized approach in patients with COPD due to underlying differences in the variability and methodology of the screening questionnaires at cut-off points to determine the depression diagnosis. However, various simplified tools can help a clinician screen out depression, and if the case is in doubt, referring to a specialist who specializes in psychiatric disorders can show beneficial effects for the patient.

Much-blooming evidence states that systemic inflammation may result in depression, and IL-6 mainly plays an essential role in human and animal models of depression [119].

### 5.9. Cardiovascular Diseases

The functional and anatomical relationship between the heart and lungs is very intricate. Any impairment that impacts one of the two organs will likely have consequences on the other. These associations are essential in COPD patients and can be of two types: (A) related pathologies that have similar risk factors, such as COPD and congestive heart failure, or smoking cigarettes and coronary artery disease (CAD), and (B) those diseases that result in the dysfunctioning of the heart to underlining primary lung diseases, such as ventricular dysfunction and secondary pulmonary hypertension due to increased intrathoracic mechanical load. Common cardiovascular diseases which are found in prevalence in COPD patients are described below.

### 5.10. Coronary Artery Disease

CAD and COPD are very prevalent diseases and share similar risk factors, such as old age, sedentary lifestyle, and smoking cigarettes. Independent of sex, age, and smoking habits, it is evident that patients with any airflow limitations are more prone to death from myocardial infarction [120]. Some results were obtained even when the history of cigarette smoke was included [121]. Some results were obtained even when the history of cigarette smoke is included [121]. Due to respiratory insufficiency, the chances of mortality due to cardiovascular ailments are higher in patients with mild COPD [105]. Clinically, a strong correlation has been found between FEV1 (impaired lung function) and cardiovascular mortality and morbidity. Independent of the status of smoking, COPD patients have a higher prevalence of fatal myocardial infarction [122].

### 5.11. Heart Failure

The shreds of evidence for the association between left ventricular congestive failure and COPD are comparatively lesser. Although some theories suggest that COPD shares a common inflammatory pathway with left ventricular congestive failure, it is clinically poorly defined how the prevalence of left ventricular function decreases in COPD patients. One study estimates that the prevalence of left ventricular congestive failure is about 20% in patients with COPD who have never had such a diagnosis [123]. The signs and symptoms of heart failure in COPD are very intricate and overlap with one another, making the diagnosis very complicated. The best way to discriminate between COPD and heart failure in COPD is the measurement of N-terminal prohormone brain natriuretic peptide (NT-proBNP) or B-type natriuretic peptide [124]. This measurement of NT-proBNP can be a valuable factor in distinguishing between decompensated heart failure and acute COPD exacerbation [125]. An overexpressed NT-proBNP plasma level correlates with poor physical activity in patients with COPD, suggesting that the defective left ventricular function may contribute to reducing the performance in the patients [126].

### 5.12. Pulmonary Arterial Hypertension (PAH)

Clinically, pulmonary arterial hypertension is not common among patients with COPD with mild to moderate stages. However, it can develop during exercise. About 50% of patients with COPD who undergo lung transplantation or lung volume reduction surgery have severe to moderate PAH [127]. The ratio between hypoxic vasoconstriction and ventilation-perfusion is higher in less severe cases of COPD than in advanced stages of COPD, where the ratio is less. Various studies suggest that the initial stages of PAH in COPD can be an injury of the endothelium by smoking cigarettes with a simultaneous downregulating of the expression of prostacyclin synthase and endothelial nitric oxide synthase and subsequently the impairment in the function of the endothelium [128].

### 5.13. Arterial Stiffness and Endothelial Function

Arterial stiffness which occurs in vascular disease is a better marker for cardiovascular events. It can be determined noninvasively by calculating the aorta's radial artery tonometry or pulse wave velocity [129]. In regular smokers and nonsmokers, arterial stiffness increases in COPD patients, and this phenomenon is neither related to the severity of the disease nor to the concentration of circulating CRP [130]. Clinically, this increase in arterial stiffness may result in systemic hypertension and increase the prevalence of cardiovascular diseases in patients with COPD [131].

## 6. Therapy Approaches in COPD

The usage of bronchodilators for the management of COPD is an important advance. It has been long acting, but the underlying mechanism for these drugs to deal with the inflammatory process is not known [132]. COPD shows heterogeneous clinical phenotypes, which leads to incongruent groups with unstable disease mechanisms or molecular pathways, leading to inconsistent approaches for the development of new therapies [133]. For COPD therapy, most known drug classes are being used in the newly approved drugs. These drugs do not target disease progression processes and mortality but address symptoms and exacerbations. Hence, a humongous requirement exists for developing therapies that target immune dysfunction and underlying inflammation [134]. After the recent elucidation of the underlying inflammatory signaling pathways in COPD, new molecular targeted drug candidates for COPD are signal-transmitting substances. Newer COPD treatment strategies are described in Figure 4 and Table 1.

### 6.1. Antioxidants

In the pathogenesis of COPD, oxidative stress plays a vital role. Antioxidants inhibit oxidative stress by scavenging reactive oxygen species (ROS), which reduces inflammation and cellular damage in the lungs [144]. In this aspect, Table 2 provides clinical testing of *N*-acetyl cysteine and other glutamines have been carried out [154].

### 6.2. Protease Inhibitors

In COPD pathophysiology, the lung's antiprotease ratio is an important aspect. Both in vitro and in vivo COPD models have shown efficacy for antiprotease therapy [155]. Selective inhibitors have been designed against matrix Metaloprotein 9 (MMP-9). These inhibitors have shown efficacy in animal models, but their effectiveness is minimal in clinical trials of COPD [156].

### 6.3. Chemokine and Cytokine Inhibitors

The levels of cytokines and chemokines like IL-1, IL-6, IL-1*β*, IL-8, and TNF-*α* increased significantly in COPD patients [157]. Inhibitors have been designed against the IL-8 receptor CXC chemokine receptor 2 (CXCR2). These inhibitors have shown positive results in animal models and clinical trials by blocking neutrophil infiltration [158] (Table 3).

### 6.4. PDE4 Inhibitors

Phosphodiesterase enzymes (PDE) metabolize the intracellular secondary messenger cAMP and cGMP. Inflammatory cells such as T-cells, eosinophils, and neutrophils have shown the expression of PDE4 in asthma and COPD [174]. Thus, inhibiting PDE4 is an effective therapeutic strategy for inflammatory respiratory diseases. PDE4 inhibitors target cAMP hydrolysis, increasing levels and activating downstream phosphorylation cascades. This reduces inflammation and relaxes the airway smooth muscles [175].

The only approved PDE4 inhibitor for treating severe COPD is roflumilast. It has been shown to improve lung function significantly and reduce the exacerbation rate in clinical trials with severe COPD [176] (Table 4).

### 6.5. Adhesion Molecule Inhibitors

Adhesion molecules are expressed on a variety of cells. They help intracellular communication via cell–cell adhesion and signal transduction [183]. An antiselectin antibody, EL246, which targets cell adhesion, has been developed. Currently, EL246 is being pursued with acute exacerbation of COPD as a therapeutic drug [184] (Table 5).

### 6.6. PPAR Agonist

The role of peroxisome proliferator-activated receptor (PPAR) signaling in regulating inflammation has been studied well. Of the various isoforms of PPAR, PPARg plays a crucial role in regulating the expression of genes involved in pathogenic conditions [192]. PPAR*γ* agonists exhibit an anti-inflammatory effect as they suppress the production of pro-inflammatory cytokines [193]. Thiazolidinediones, one of the PPAR*γ* agonists, have reduced lung inflammation in in vivo studies [194]. In cigarette smoke-induced emphysema, thiazolidinediones treatment was shown to reverse the emphysema [195].

## 7. Conclusions and Prospects

Many comorbidities are present with COPD, which is associated with inaccuracy in death. So, all causes of death must be the prime endpoint for any further studies to evaluate the therapy of COPD. However, the ongoing revolution of COPD health studies, including all causes of mortality, can provide conclusive data for long-acting b2-agonists and inhaled corticosteroids in combination or individually. It is essential to consider COPD as a multicomponent disease [196] with severe comorbidities, such as lung cancer, cardiovascular diseases, and systemic and pulmonary inflammation. Recently, orally administered broad-spectrum anti-inflammatory therapies have been in clinical development, but they appear to have remarkable side effects, so inhaled drugs should be developed for future perspectives. Another approach should be to develop a drug that reverses the resistance of corticosteroids, which is supposed to be a massive barrier to the therapies [197]. In the future, a clear understanding of the molecular mechanism behind corticosteroid resistance may lead to new therapeutic approaches.

Another future area of research should consider COPD and various comorbidities, including osteoporosis, diabetes, and cardiac disease, as a disease of accelerated aging. Molecular pathways behind aging are very well understood and reveal many novel drug targets as interventions, including peroxisome proliferator-activated-*γ* coactivator 1*α* and antiaging molecules sirtuin 1 [198]. This review has discussed different types of diagnostic biomarkers used to detect and confirm COPD. These biomarkers help identify the diseased population and aid us in redefining the disease classification. COPD pathogenesis majorly consists of overexpression of systemic inflammation markers and signaling pathways. Thus, determining these markers is one of the imperative and crucial directions in improving the diagnosis and management of COPD.

## Figures and Tables

**Figure 1:** Risk factors of COPD.

**Figure 2:** List of biomarkers used in the diagnosis of COPD. ECB, exhaled blood condensate; LPP, lipid peroxidation product; and Pro-ISR, pro-inflammatory signaling receptor.

**Figure 3:** Comorbidities with COPD.

**Figure 4:** Molecular targets for newer COPD treatment strategies [14].

**Table 1:** Pro-inflammatory signaling pathway inhibitors for COPD.

S. no.	Inhibitor/drug	Mechanism/effect	Clinical progress	References
1	RV568	P38MAPK pathway inhibitor	No effect (NCT01475292) (NCT01661244)	[135]

2	Nemiralisib (GSK2269557)	PI3K inhibitor	28 Days treatment (NCT02294734) 84 Days treatment (NCT02522299)	[136]

3	RV1729	PI3K inhibitor	Phase I Trial, limited efficacy (NCT02140346)	[136, 137]

4	VIP (vasoactive intestinal peptide)	Increases cAMP, adenylate cyclase, and phospholipase C	3 Months inhaled treatment (NCT00464932)	[138, 139]

5	Adenosine A2A receptor (UK-432097)	cAMP enhancer	No effect (NCT00430300)	[140, 141]

6	AZD1981	Prostaglandin D_2_ receptor inhibitor	No effect (NCT00690482)	[142]

7	Bimosiamose	Selectins inhibitor	28 Days inhalation treatment (NCT01108913)	[143]

**Table 2:** Antioxidants and protease inhibitors for COPD.

S. no.	Inhibitor/drug	Mechanism/effect	Clinical progress	References
1	*N*-acetyl cysteine (NAC)/glutamines	Oxidative stress suppressor	Clinical trials are going on. Effective in high-risk patients (NCT01136239) (NCT00184977)	[145, 146]

2	SOD/GPx	ROS reducer	Established in animal models. Clinical trials underway	[147]

3	Sulforaphane	ROS and RNS reducer	4 Weeks clinical study, no effect (NCT01335971)	[148]

4	Resveratrol	Activator of SIRT1	12 Weeks of clinical study done (NCT03819517)	[149]

5	SRT1720	Activator of SIRT1	Established in animal model	[150]

6	AZD1236	Anti MMP-9 and MMP-12	6 Weeks clinical study. Results not statistically significant	[151]

7	Sivelestat (ONO-5046)	Protection from NE-mediated lung damage	Clinically approved in Japan for ALI and ARDS	[152]

8	AZD9668	Protection from NE-mediated lung damage	12 Weeks clinical study with budesonide. No effect	[153]

**Table 3:** Cytokine and chemokine receptor inhibitors for COPD.

S. no.	Inhibitor/drug	Mechanism/effect	Clinical progress	References
1	Tocilizumab	IL-6 inhibitor	Clinical trials need further study	[159]

2	Canakinumab	IL-1*β* inhibitor	Phase I/II RDBPCES	[160]

3	Infliximab	TNF-*α* inhibitor	No effect (NCT00056264)	[161–163]

4	Etanercept	TNF-*α* inhibitor	90 Days treatment of COPD (NCT00789997)	[164]

5	AZD4818	CCR1 inhibitor	No effect (NCT00629239)	[165]

6	AZD2423	CCR1 inhibitor	A study completed statistical analysis not released (NCT012115279)	[166]

7	Navarixin (MK-7123)	CXCR2 inhibitor	6 Months of study. Improvement in FEV1 (NCT01006616) (NCT00441701)	[166, 167]

8	AZD5069	CXCR2 inhibitor	4 Weeks treatment (NCT01233232)	[166]

9	BIIL 284	LTB4 receptor inhibitor	Clinical study done (NCT02249247) (NCT02249338)	[168]

10	Zileuton	5-LO inhibitor	No effect in treatment (NCT00493974)	[169]

11	Mepolizumab	IL-5 inhibitor	26–52 Weeks treatment (NCT02105948, NCT01463644, NCT02105961)	[170]

12	Benralizumab	IL-5R*α* inhibitor	No effect (NCT01227278)	[171]

13	Lebrikizumab	IL-13 inhibitor	Decline in COPD exacerbation and lung function (NCT02546700)	[172, 173]

**Table 4:** cAMP and cGMP phosphodiesterase inhibitor for COPD.

S. no.	Inhibitor/drug	Mechanism/effect	Clinical progress	References
1	Roflumilast	PDE4 inhibitor	US-FDA approved drug	[177, 178]

2	GSK-256066	PDE4 inhibitor	4 Weeks inhaled treatment (NCT00549679)	[179]

3	CHF6001	PDE4 inhibitor	Clinical testing going on (NCT01730404)	[180]

4	Tadalafil	PDE5 inhibitor	Approved for pulmonary arterial hypertension 12-week treatment (NCT01197469)	[181]

5	RPL554	PDE3/PDE4 inhibitor	Being investigated as an adjunct (NCT02542254)	[182]

**Table 5:** Other drugs for COPD.

S. no.	Inhibitor/drug	Mechanism/effect	Clinical progress	References
1	Eleuquin (EL246)	Cell adhesion inhibitor	Under predevelopment by LigoCyte	[185]

2	BIBW 2948	EGFR internalization reducer	4 Weeks treatment (NCT00423137)	[186]

3	Bosentan	Endothelin receptor inhibitor	18 Months treatment (NCT02093195)	[187, 188]

4	Solithromycin	Macrolide antibiotic	Early termination of the trial (NCT02628769)	[189]

5	Thiazolidinediones	PPAR*γ* agonists	10 Months treatment (NCT00103922)	[190, 191]

## Data Availability

The data that support this study's findings are available in this article.
